# Diversity Evolutionary Policy Deep Reinforcement Learning

**DOI:** 10.1155/2021/5300189

**Published:** 2021-08-03

**Authors:** Jian Liu, Liming Feng

**Affiliations:** ^1^School of Information and Control Engineering, China University of Mining and Technology, Xuzhou 221116, China; ^2^Engineering Research Center of Intelligent Control for Underground Space, Ministry of Education, China University of Mining and Technology, Xuzhou 221116, China

## Abstract

The reinforcement learning algorithms based on policy gradient may fall into local optimal due to gradient disappearance during the update process, which in turn affects the exploration ability of the reinforcement learning agent. In order to solve the above problem, in this paper, the cross-entropy method (CEM) in evolution policy, maximum mean difference (MMD), and twin delayed deep deterministic policy gradient algorithm (TD3) are combined to propose a diversity evolutionary policy deep reinforcement learning (DEPRL) algorithm. By using the maximum mean discrepancy as a measure of the distance between different policies, some of the policies in the population maximize the distance between them and the previous generation of policies while maximizing the cumulative return during the gradient update. Furthermore, combining the cumulative returns and the distance between policies as the fitness of the population encourages more diversity in the offspring policies, which in turn can reduce the risk of falling into local optimal due to the disappearance of the gradient. The results in the MuJoCo test environment show that DEPRL has achieved excellent performance on continuous control tasks; especially in the Ant-v2 environment, the return of DEPRL ultimately achieved a nearly 20% improvement compared to TD3.

## 1. Introduction

Reinforcement learning [1, 2], as an important branch of machine learning [3, 4], has always been a research hotspot. Reinforcement learning constantly improves its policy by interacting with the actual environment, so that the policy can get the maximum cumulative return in the current environment. In recent years, deep learning has exerted more and more influence on various research fields. The combination of deep learning and reinforcement learning produces a variety of deep reinforcement learning algorithms. Deep reinforcement learning can be divided into three types: value-based deep reinforcement learning [5–7], policy-based deep reinforcement learning [8], and deep reinforcement learning based on actor-critic structure [9–11].

Value-based deep reinforcement learning methods estimate the value function through a neural network and use the value function output by the neural network to guide the agent to choose policies, such as deep Q network (DQN) algorithm [12]. Policy-based deep reinforcement learning methods can parameterize policies and achieve policy optimization through learning parameters, so that the agent can obtain the largest cumulative return, such as deterministic policy gradient (DPG) algorithm [5]. This type of algorithm has good performance when dealing with high-dimensional continuous space problems, but it is easy to cause gradient disappearance in the process of policy update and then fall into the local optimal solution problem [8]. Deep reinforcement learning methods based on actor-critic structure combine value-based and policy-based methods to learn policies while fitting value functions, such as deep deterministic policy gradient (DDPG) algorithm. Actor network parameters are trained according to the value function output by the critic network, and the critic network parameters are updated in a single step using the time difference (TD) method. Although the actor-critic-based methods have the advantages of both value-based and policy-based methods, they also inherit the shortcomings of the policy gradient algorithm; that is, the policy update falls into a local optimal solution due to the disappearance of the gradient.

The DDPG algorithm combines the ideas of DQN [12] and DPG [5] to solve tasks under continuous action. As an off-policy actor-critic algorithm, DDPG can be trained with historical data through experience playback pool, which greatly improves the utilization of samples and achieves better results in continuous action tasks. Subsequently, inspired by double DQN [13], twin delayed deep deterministic policy gradient algorithm (TD3) [10] on the basis of DDPG simultaneously uses two critic networks to fit the state action value function. And it takes the minimum value of the two target network outputs as the final estimate. TD3 solves the problem of overestimation of the DDPG median function and improves the stability of the agent. However, since DDPG and TD3 both use a similar way to the policy-based algorithms when updating the policy, they also rely on the gradient information for updating policy, which undoubtedly suffers from the vanishing gradient problem during the update process. By adding a small amount of random noise to the policy output by the neural network, the influence of the disappearance of the gradient on the policy update can be alleviated to a certain extent. For example, NoisyNets [14] enhance the exploration ability of the algorithm by directly adding random noise to the parameters of the neural network. However, since the influence of random noise on the policy is random and nondirectional, the effect of this method is limited. The combination of policy gradient and deep learning can be applied to complex and challenging tasks such as game simulation [15], robot control [16], and dialogue system [17]. However, when the policy gradient methods are applied to the continuous control filed, there still exists a basic problem, that is, the local optimal problem caused by the disappearance of gradient in the updating process. Tessler et al. [8] put forward that the generation model can be used to learn policies. In this way, although local optimal problem can be avoided, the difficulty of algorithm training is increased.

Evolutionary policy has been used as a nongradient optimization algorithm for decades and performs well in some reinforcement learning benchmark environments. Compared with gradient optimization, the evolution policy is simpler to implement, uses fewer hyperparameters, does not require gradient information, is easier to expand in a distributed environment, and is less affected by sparse rewards. Wierstra et al. [18] proposed Natural Evolution Policies (NES), which optimizes the policy by searching for the distribution of parameters and uses natural gradients to update the distribution in the direction of higher fitness. Inspired by the NES, Tim et al. [19] used the NES as a nongradient black box optimizer to find the optimal policy parameters. Khadka and Tumer [20] proposed evolutionary reinforcement learning (ERL) by effectively combining the evolutionary algorithm based on population with DDPG. Based on ERL, Pourchot and Sigaud [21] combined the cross-entropy method (CEM) with reinforcement learning and proposed CEM-RL method, which further improved the performance of the algorithm.

At present, most of the algorithms that combine reinforcement learning and evolutionary policy only make use of the cumulative return information of policies in each generation population but do not make full use of the distance information of policies between different generations. Effectively increasing the distance between policies of different generations is conducive to the generation of diverse policies for future generations and can improve the exploration of the environment by the reinforcement learning agent. Simultaneously, compared with the single policy, the diverse policies can effectively reduce the risk of falling into the local optimal solution in the updating process. Therefore, in this paper, a diversity evolutionary policy deep reinforcement learning (DEPRL) algorithm is proposed. DEPRL uses maximum mean discrepancy (MMD) to measure the distance between different policies. In the contemporary population, some policies maximize the cumulative return while maximizing the distance from the previous generation policy during the gradient update process. In the process of population evolution, the distance information and cumulative return of the policy are taken as the fitness of the population. The difference between the new generation policy and the previous generation policy is enlarged on the basis of ensuring the higher cumulative return of the new generation policy. By diversifying the policies in the population, DEPRL reduces the risk that the algorithm will fall into local optimum due to the disappearance of gradient in the process of updating and improves the exploration efficiency of agents. Finally, the effectiveness of DEPRL in continuous action task is verified by MuJoCo simulation environment.

The remainder of this paper is organized as follows. The next section describes the related works of DEPRL method.  Section 3 represents the framework and details of DEPRL method. Then, in Section 4, a series of comparison experiments on MuJoCo test environment are conducted. The final section provides our concluding remarks and points out our future work orientation.

## 2. Related Works

### 2.1. Markov Decision Process (MDP)

In reinforcement learning, the interaction process between reinforcement learning agents and the environment can be represented by Markov decision process (MDP). MDP can be represented by a tuple *M*=(*S*, *A*, *R*, *P*^*t*^, *γ*), where *S* is the state space, *A* is the action space, *R* is the reward function, *P*^*t*^ is the state transition probability, and *γ* ∈ [0 ~ 1] is the discount factor. When the agent interacts with the environment, the way of choosing an action is called an action policy. Generally, the action policy can be a random policy or a deterministic policy. The random policy *π* is a probability value, which represents the probability that the agent chooses different actions from the action space in the state *S*, and the deterministic policy *π*_*η*_ represents the choice of a certain action in the state *S*. In each time step, the agent observes the current state *s*_*t*_ ∈ *S* according to the environment and chooses action *a*_*t*_ ~ *π*(*s*_*t*_) according to the policy to get the reward *r*_*t*_=*r*(*s*_*t*_, *a*_*t*_) of the environment feedback. Subsequently, the agent enters the next state according to the state transition probability *P*^*t*^. The goal of reinforcement learning is to train the agent so that the agent finds an optimal policy *π*^*∗*^ that can obtain the largest cumulative return.

### 2.2. Cross-Entropy Method (CEM)

Evolutionary algorithms update the population by managing a finite number of individuals and generating new individuals near the previous elite sample. Some evolutionary algorithms are temporary optimization methods based on heuristics, such as genetic algorithm (GA) [22]. And the other part is based on the distribution algorithm that estimates the elite sample, such as estimation of distribution algorithms (EDA) [23, 24]. Cross-entropy method (CEM) is a simple EDA algorithm. Suppose that the total number of individuals in the population is *K*, where the total number of elite individuals is fixed at a certain value *K*_*e*_, which is usually set to half of the total number of individuals in the population. After evaluating all the individuals in the population, the first *K*_*e*_ outstanding individuals are used to calculate the new mean and variance of the population. Then, additional variance is added to prevent premature convergence, and the next generation is sampled from the new population. A new distribution is obtained by adding Gaussian noise *ε* around the average value *μ* of the distribution, so that each individual (*x*_*i*_)_*i*=1,…,*K*_ is sampled from this new distribution, that is, *x*_*i*_ ~ *𝒩*(*μ*, Σ), where Σ represents the current covariance matrix. By calculating the fitness of these newly generated individuals related to specific problems, CEM uses the best performing *K*_*e*_ individuals (*z*_*i*_)_*i*=1,…,*K*_*e*__ to update the distribution parameters.

### 2.3. Neural Networks

In recent years, many neural networks, such as extreme learning machine (ELM) [25], probabilistic neural network (PNN) [26], and deep neural networks (DNN) [27], have been proposed and applied in many research fields. For example, Yi et al. [26] proposed a self-adaptive probabilistic neural network (SaPNN) method for transformer fault diagnosis problem. SaPNN can select the best spread self-adaptively all the time and always get the best prediction accuracy. To improve the accuracy and usefulness of target threat assessment in the aerial combat, Wang et al. proposed Elman-AdaBoost strong predictor [28] and multiple wavelet function wavelet neural networks (MWFWNN) [29] to solve threat assessment. Elman-AdaBoost strong predictor uses the Elman neural network as a weak predictor and obtains a strong predictor composed of multiple Elman neural network weak predictors through the Elman-AdaBoost algorithm. In [29], a wavelet mother function selection algorithm was proposed with minimum mean squared error and used to construct MWFWNN network. Cui et al. [30] proposed a novel method that used convolutional neural network (CNN) to improve the detection of malware variants. They converted the malicious code into grayscale images and used CNN to identify and classify the images.

Neural networks can also be applied to reinforcement learning. Traditional reinforcement learning is limited to small action space and sample space, which are generally discrete. However, more complex and more realistic tasks often have a large state space and continuous action space. When the input data is image or sound, it usually has a very high dimension, which is difficult for traditional reinforcement learning to deal with. Deep reinforcement learning is to combine the high-dimensional input of deep neural networks with reinforcement learning. Deep Q network (DQN) [12] can be regarded as the beginning of the successful combination of the two. It uses a deep network to represent the value function. Based on Q-learning in reinforcement learning, it provides target values for the deep network and constantly updates the network until convergence. After that, many deep reinforcement learning algorithms have been proposed, such as double DQN [13], DPG [5], and TD3 [10].

### 2.4. Twin Delayed Deep Deterministic Policy Gradient Algorithm (TD3)

Both DDPG and TD3 are off-policy reinforcement learning algorithms based on the actor-critic structure. DDPG is easy to cause the problem of overestimation of value function, which affects the stability of algorithm. To mitigate the negative effects of overestimation, TD3 uses both critic networks to estimate the state action values and takes the minimum value of the two target network outputs as the final estimate.

In order to make the parameters of actor and critic networks updated stably, TD3 makes the updating frequency of network parameters of actor network lower than that of critic network during the training process. TD3 also adds random noise to the action output by the target policy, which not only improves the agent's exploration ability, but also fits the state action value of a small area around the target action. TD3 makes the value function learned by critic network smoother in the action dimension. Since the update direction of actor network parameters is affected by the value function learned from the critic network, the policy learned from actor network also tends to be smoother in the action dimension. By adding random noise, TD3 improves the stability of the agent during training process. The calculation formula of the action value of the target state in TD3 is as follows:

(1) $$\begin{array}{c} y\left(r,s^{\prime }\right)=r+\gamma \underset{i=1,2}{\min}Q_{\phi_{i}}\left(s^{\prime },\pi_{\theta }\left(s^{\prime }\right)+\varepsilon \right),\\ \varepsilon ∼\text{clip}\left(N\left(0,\sigma \right),-c,c\right). \end{array}$$

## 3. Methods

### 3.1. Diversity Evolutionary Policy Deep Reinforcement Learning (DEPRL)

The objective function of DEPRL mainly includes the objective function of critic network and actor network. To mitigate the impact of overestimation of the value function, critic network takes the minimum value of the two target network outputs to calculate the final target value. Assuming that *θ*_1_ and *θ*_2_ represent the estimated network parameters of the two critic networks, *θ*_*t*arg,1_ and *θ*_*t*arg,2_ represent target network parameters of the two critic networks. Then, the update process of the critic networks in DEPRL is shown in Figure 1. The target value of state action under time steps *t* is

(2) $$\begin{array}{c} Y\left(s_{t},a_{t}\right)=r+\gamma \underset{i=1,2}{\min}Q_{\theta_{t\arg,i}}\left(s_{t+1},\pi_{\phi }\left(s_{t+1}\right)\right), \end{array}$$

where *r* is the reward to the environment, *Q*_*θ*_*t*arg,*i*__(*s*_*t*+1_, *π*_*ϕ*_(*s*_*t*+1_)) represents the target network output value of the *i*-th critic network, *ϕ* represents the network parameters of the actor network, and *γ* is the discount factor. Assume that *Q*_*θ*_*i*__(*s*_*t*_, *a*_*t*_) represents the estimated value output by the *i*-th estimation network under the number of time steps *t*, and then the objective function of critic network can be written as

(3) $$\begin{array}{c} J_{Q}\left(\theta_{i}\right)=E_{\left(s_{t},a_{t}\right)∼D}\left[\frac{1}{2}{\left(Q_{\theta_{i}}\left(s_{t},a_{t}\right)-Y\left(s_{t},a_{t}\right)\right)}^{2}\right]. \end{array}$$

Therefore, the estimated network parameters *θ*_1_ and *θ*_2_ can minimize the objective function *J*_*Q*_(*θ*_*i*_) through gradient descent. That is, gradient descent is used to minimize the mean square error between the estimate and the target value:

(4) $$\begin{array}{c} \theta_{1}⟵\theta_{1}-\alpha \nabla_{\theta_{1}}\frac{1}{2}{\left(Q_{\theta_{1}}\left(s_{t},a_{t}\right)-Y\left(s_{t},a_{t}\right)\right)}^{2},\\ \theta_{2}⟵\theta_{2}-\alpha \nabla_{\theta_{2}}\frac{1}{2}{\left(Q_{\theta_{2}}\left(s_{t},a_{t}\right)-Y\left(s_{t},a_{t}\right)\right)}^{2}, \end{array}$$

where *α* represents the update step size. In the process of gradient updating, the target network parameters *θ*_*t*arg,1_ and *θ*_*t*arg,2_ are kept constant to ensure the stability of updating.

After the estimated network parameters are updated, the parameters of the target network are updated by soft update method. The formula is as follows:

(5) $$\begin{array}{c} \theta_{t\arg,1}⟵\tau \theta_{1}+\left(1-\tau \right)\theta_{t\arg,1}, \end{array}$$

(6) $$\begin{array}{c} \theta_{t\arg,2}⟵\tau \theta_{2}+\left(1-\tau \right)\theta_{t\arg,2}, \end{array}$$

where *τ* is the coefficient of soft update method. For the parameter *ϕ* of actor network, the gradient update direction is to maximize the distance between the current policy and *π*_*η*_ while maximizing the cumulative return. The distance between *π*_*η*_ and the current policy can be calculated by using the square of the maximum mean discrepancy (MMD).

Given samples *x*_1_,…, *x*_*n*_ ~ *P* and *y*_1_,…, *y*_*m*_ ~ *G*, the square of the MMD can be estimated only from the sample of the distribution. Then, the square of MMD between distribution *P* and *G* can be written as

(7) $$\begin{array}{c} {\text{MMD}}^{2}\left(\left\{x_{1},\ldots ,x_{n}\right\},\left\{y_{1},\ldots ,y_{m}\right\}\right)=\frac{1}{n^{2}}\sum_{i,i^{\prime }}k\left(x_{i},x_{i^{\prime }}\right)-\frac{2}{nm}\sum_{i,j}k\left(x_{i},y_{j}\right)+\frac{1}{m^{2}}\sum_{j,j^{\prime }}k\left(y_{j},y_{j^{\prime }}\right), \end{array}$$

where *k*(·, ·) is the kernel function. Here, Gaussian kernel is used in DEPRL, that is,

(8) $$\begin{array}{c} k\left(x_{i},x_{i^{\prime }}\right)=\exp\left(-\frac{{\left\|x_{i}-x_{i^{\prime }}\right\|}^{2}}{2\sigma^{2}}\right),\;\sigma >0, \end{array}$$

where *σ* is standard deviation. Record the square of MMD between policy *π*_*η*_ and policy *π*_*ϕ*_ as *D*_MMD_(*π*_*η*_, *π*_*ϕ*_), and the formula is as follows:

(9) $$\begin{array}{c} D_{\text{MMD}}\left(\pi_{\mu },\pi_{\phi }\right)={\text{MMD}}^{2}\left(\pi_{\mu }\left(\cdot |s\right),\pi_{\phi }\left(\cdot |s\right)\right)\;s∼D, \end{array}$$

where *D* is the experience pool.

To sum up, the objective function of actor network only considering the maximum cumulative return is

(10) $$\begin{array}{c} J_{\pi }\left(\phi \right)=E_{s∼D,a∼\pi_{\phi }\left(\times |s\right)}\left[Q_{\theta_{1}}\left(s,a\right)\right]. \end{array}$$

When *D*_MMD_(*π*_*η*_, *π*_*ϕ*_) that satisfies the gradient update requirement is obtained, the objective function of the actor network can be written as

(11) $$\begin{array}{c} J_{\text{MMD}}\left(\phi \right)=E_{s∼D,a∼\pi_{\phi }\left(\cdot |s\right)}\left[Q_{\theta_{1}}\left(s,a\right)\right]+\beta E_{s∼D}\left[{\text{MMD}}^{2}\left(\pi_{\mu }\left(\cdot |s\right),\pi_{\phi }\left(\cdot |s\right)\right)\right], \end{array}$$

where *β* > 0 is the weighting factor. The number of actors that only consider cumulative returns is recorded as *K*_1_, and then the number of actors that maximize *D*_MMD_(*π*_*η*_, *π*_*ϕ*_) at the same time is *K*/2 − *K*_1_.

### 3.2. The Framework of DEPRL

In CEM-RL method, the total number of individuals in the population is set to *K*. The mean *μ* and covariance matrix Σ of the policy parameter distribution are obtained by random initialization. According to the covariance matrix and the mean value, *K* parameters are extracted from the distribution as the parameters of actor network in the population. The actor network with half of the total number of individuals in the population is randomly selected for gradient update according to the value function output from critic network. The goal is to maximize the cumulative return of the actor network's corresponding policy. The critic network that guides actor network gradient updates throughout the process is the same; that is, half of the actors in the population use the same critic network to guide updates. In a population, the data generated by the interaction between the actor and the environment is stored in the experience pool and is used to train the critic network. By evaluating the cumulative returns of the policies corresponding to all actors in the population after gradient updating, the policies ranked in the top half of the cumulative returns are selected as the elite sample. The number of the elite sample *K*_*e*_ is usually set to *K*_*e*_=*K*/2. Finally, according to the parameters of contemporary elite samples, *μ*_new_ and Σ_new_ of the new generation actor network parameter distribution are generated.

The framework of DEPRL algorithm is shown in Figure 2. Assume that the corresponding policy of Actor_*μ*_ composed of elite sample parameters is *π*_*η*_. When the critic network guides the next generation policy update, it needs to maximize the MMD between a part of policies and *π*_*η*_. By increasing the diversity of descendant policies, more space is explored, and the probability of the algorithm falling into the local optimal solution is reduced. When selecting the elite sample, not only the cumulative return of each policy should be considered, but also the MMD between each policy and *π*_*η*_ should be considered. In the population, the updated new policy is first sorted according to the cumulative return from high to low, and the policies with cumulative return ranked between 2 and *K*/2 greater than *πμ* cumulative return are taken out, and the MMD values between these policies and *π*_*η*_ are calculated, and reorder the MMD value from largest to smallest. In the population, the updated new policy is first sorted according to the cumulative return from high to low. Then, the policies in which the cumulative return is between 2 and *K*/2 greater than the cumulative return of *π*_*η*_ are taken out. Finally, the MMD values between these policies and *π*_*η*_ are calculated. These policies are reordered in descending order of MMD value.

Use MMD as the standard to select policies that is quite different from *πμ* among contemporary policies, which helps transfer the diversity policy to the next generation distribution. The new generation policy generated by sampling in the new distribution is quite different from the old policy, which makes the trajectory of the new generation policy more diversified and can increase the exploration space. In order to reduce the amount of calculation when calculating the new distribution parameters, Σ is constrained to be a diagonal matrix. The update formulas of the new distribution parameters *μ*_new_ and Σ_new_ are as follows:

(12) $$\begin{array}{c} \mu_{\text{new}}=\sum_{i=1}^{K_{e}}\lambda_{i}z_{i}, \end{array}$$

(13) $$\begin{array}{c} \Sigma_{\text{new}}=\sum_{i=1}^{K_{e}}\lambda_{i}\left(z_{i}-\mu_{\text{old}}\right){\left(z_{i}-\mu_{\text{old}}\right)}^{T}+\varepsilon , \end{array}$$

where *λ*_*i*_ represents the weight of the parameter corresponding to the *i*-th elite policy in the population, and *ε* is the Gaussian noise. *λ*_*i*_ can be defined as

(14) $$\begin{array}{c} \lambda_{i}=\frac{\left(\log\left(1+K_{e}\right)/i\right)}{\sum_{i=1}^{K_{e}}\left(\log\left(1+K_{e}\right)/i\right)}. \end{array}$$

The above formula indicates that the higher the ranking of the parameters corresponding to the elite policy, the greater the value of a *λ*_*i*_.

To sum up, the update process of DEPRL can be simply summarized as follows: (1) the parameter distribution of the initialization policy is *N* (*μ*_0_, *∑*_0_); (2) *K* group policies are randomly selected corresponding to *K* group parameters from the distribution; (3) gradient updating is performed by randomly selecting *K*/2 policy; (4) the fitness of the corresponding policy under the *K* set of parameters is calculated; (5) the parameters corresponding to the current elite policy are used to calculate the parameter distribution (*μ*, *∑*) of the next generation policy, as shown in equations (12) and (13); (6) whether the parameter distribution of the contemporary policy meets the requirements is determined; if so, stop updating; if not, repeat step (2).

The pseudocode of DEPRL algorithm is shown in Algorithm 1.

## 4. Results and Analysis

### 4.1. Experiment Settings

In this section, we use the MuJoCo test environment implemented in OpenAI Gym [31] to evaluate the performance of the proposed algorithm and comparison Algorithms. Gym is a basic platform for testing deep reinforcement learning algorithms provided by OpenAI. It provides a large number of simple interfaces for the training of the agent, greatly simplifies the interaction process between the agent and the environment, and facilitates related researchers to implement deep reinforcement learning algorithms and test the performance of deep reinforcement learning algorithms.  Figure 3 shows the corresponding status screens of the four tasks in the MuJoCo test environment.  Table 1 describes the state dimension and action dimension of the four tasks in the MuJoCo test environment, as well as specific task goals. According to the state dimension and action dimension information provided by MuJoCo, it is convenient to design the corresponding neural network for learning. The version of OpenAI Gym used in the experiment is 0.17.3, and the version of MuJoCo is 2.0.

Experiment settings are set up as follows:

1. We chose to compare TD3, multiactor TD3, CEM, and CEM-TD3 to verify the superiority of the proposed DEPRL. The common superparameter settings of the five algorithms are the same as shown in Table 2, and the total numbers of population individuals and elite individuals of CEM-TD3 and DEPRL are the same, 10 and 5, respectively. When DEPRL calculates *D*_MMD_, the data size *M* extracted from the experience pool is 600, the number of Gaussian kernel function *m* = *n* = 5, and the value of *K*_1_ is 4. The weighting factor *β* in the objective function *J*_MMD_ is 0.2 in the Ant-v2 environment, and 0.1 in all other test environments.
2. In order to make a fair comparison between different algorithms, we combined CEM and TD3 to form CEM-TD3 algorithm for experiment. And the network structure used by CEM to represent policies is consistent with that of DEPRL, CEM-TD3, multiactor TD3 and TD3. Multiactor TD3 is a variant of TD3. Compared with TD3, multiactor TD3 has multiple actors. The experience data generated by the interaction between multiple actors and the environment are sent to the experience pool together, and the critic remains unchanged. In the experiment, the number of actors in multiactor TD3 is set to 5, and the total number of gradient updates of critic and actor in multiactor TD3, CEM-TD3, and DEPRL is the same.
3. We selected four environments HalfCheetah-v2, Hopper-v2, Walker2d-v2, and Ant-v2 for comparison, and the details of the test environment are shown in Table 1. The experimental results are shown in Figure 4, where the horizontal axis represents the number of time steps, and the vertical axis represents the cumulative return value of a round in the evaluation stage. During the training process, the performance of the current algorithm is evaluated every 1000 steps. Each algorithm was repeated with five different random seeds in different test environments. When drawing the reward curve, the sliding window size is set to 100. The curve part and shaded part in the figure represent the mean value and the standard deviation of the accumulated return value under multiple random seeds, respectively. We also present the mean and standard deviation of the cumulative return per turn in different MuJoCo tasks. The results can be found in Table 3.

### 4.2. Analysis of Experimental Results

1. As can be seen from Figure 4, DEPRL performs best overall in the test environment and also performs best in the environment with higher state dimension and action dimension, such as Ant-v2 and Walker2d-v2. CEM performs worst overall and learns few effective policies in environments with higher state and action dimensions. Therefore, it can be shown that both the sample utilization and learning rate of CEM are significantly lower than those of other algorithms based on single-step update.
2. In order to explore whether the improvement of DEPRL effect is due to the adoption of multiactor structure, we tested the influence of multiactor structure on the algorithm. Compared with the traditional actor-critic structure, the training data used by the critic in the multiactor structure is generated by the interaction between multiple actors and the environment. By comparing the reward curves of TD3, multiactor TD3, and DEPRL in Figure 4, it can be found that the reward curve of multiactor TD3 is only slightly higher than that of TD3 based on the traditional actor-critic structure. Therefore, it can be explained that the multiactor structure does not improve the algorithm much. In the Hopper-v2 training environment, multiactor TD3 began to oscillate when the cumulative return of the policy reached about 3200 and could not learn a better policy, while DEPRL with the same multiactor structure could get about 3600 cumulative returns. By comparing the reward curves among TD3, multiactor TD3, and DEPRL, it can be shown that the performance improvement of DEPRL does not simply depend on the multiactor structure.
3. To explore the benefits of DEPRL in encouraging offspring diversity, we compared it with CEM-TD3, which only uses cumulative returns as a policy learning goal. CEM-TD3 also uses multiactor structure, and the total number of population individuals and the number of elite individuals is set the same as DEPRL. It can be seen from Figure 4 that the reward curve of DEPRL is significantly higher, and the reward curve of CEM-TD3 gradually levelled off in the second half due to the decline of exploration ability. Except for the Hopper-v2 test environment, DEPRL still maintained a relatively high growth trend in the second half of the reward curve.
4. As can be seen from Table 3, the DPERL algorithm has the highest mean cumulative return of all the algorithms. The CEM algorithm performs the worst, which once again demonstrates that CEM, as a turn update algorithm with no experience replay, could not learn effective strategies. Compared with TD3 and multiactor TD3 algorithms, DPERL and CEM-TD3 algorithms have higher average cumulative returns, which is due to the addition of evolutionary strategy into DPERL and CEM-TD3 algorithms. Compared with the CEM-TD3 algorithm, the DPERL algorithm achieves better results, because it increases exploration by encouraging the generation of diversity strategies in the offspring. In addition, in the Hopper-v2, HalfCheetah-v2, and Ant-v2 test environments, DPERL has smaller standard deviations than TD3, multiactor TD3, and CEM-TD3 algorithms, which indicates that DPERL algorithm has more stable results than the other three algorithms. To some extent, this also shows that DPERL algorithm can explore more effective strategies.

The above results clearly show that DEPRL improves the exploration ability of reinforcement learning agents and, to some extent, reduces the risk of policy updating falling into local optimum due to the disappearance of gradient.

## 5. Conclusions and Discussions

In this paper, we propose the DEPRL algorithm, which combines CEM and TD3 to measure the distance between different policies through MMD method. Some contemporary policies maximize the cumulative return while maximizing the distance between them and the previous generation policies and obtain policies with large differences to increase the scope of exploration. In the course of evolution, combining the cumulative return of a contemporary policy with the distance between the previous generation's policy as fitness helps the next generation's policy have more diversity based on a higher cumulative return. By combining TD3 with gradient updating and CEM without gradient updating, DEPRL can reduce the risk of policy updating falling into local optimal solution due to gradient disappearance by encouraging the generation of diversified policies in the offspring. By comparing DEPRL with CEM-RL, TD3, CEM, and multiactor TD3 in MuJoCo test environment, the experimental results show that DEPRL achieves more effect without increasing the number of update steps.

In DEPRL, we use an estimation of distribution algorithm to estimate the distribution of the elite samples and then select the elite samples that meet certain conditions to improve the diversification of the elite strategy. Except for estimation of distribution algorithms, some of the most representative computational intelligence algorithms can be used to reinforcement learning. Monarch butterfly optimization (MBO) [32] algorithm generates offspring by migration operator, which can be adjusted by the migration ratio of monarch butterflies. It is followed by tuning the positions for other butterflies by means of butterfly adjusting operator. In reinforcement learning, MBO can adjust the selection of elite samples in the global scope to avoid the loss of potential elite samples. In earthworm optimization algorithm (EWA) [33], the offspring are generated through Reproduction 1 and Reproduction 2 independently, and then, the weighted sum of all the generated offspring is used to get the final earthworm for next generation. Reproduction 1 generates only one offspring by itself that is also special kind of reproduction in nature. Reproduction 2 is to generate one or more than one offspring at one time. EWA can be used to replicate elite samples to ensure the high efficiency of elite strategies in reinforcement learning and speed-up learning. In elephant herding optimization (EHO) [34], the elephants in each clan are updated by its current position and matriarch through clan updating operator. It is followed by the implementation of the separating operator, which can enhance the population diversity at the later search phase. EHO is an appropriate way to increase the diversity of a population. Not only can it be used to eliminate bad reinforcement learning strategies, but it can also be used to add new strategies that did not exist before. Exploration is a vital part of reinforcement learning. Exploratory algorithms in computational intelligence algorithms can provide meaningful guidance for reinforcement learning. For example, slime mould algorithm (SMA) [35] uses adaptive weights to simulate the process of producing positive and negative feedback of the propagation wave of slime mould based on bio-oscillator to form the optimal path for connecting food with excellent exploratory ability and exploitation propensity. According to the moth's phototaxis and Levy flight characteristics, moth search (MS) [36] algorithm can do exploitation and exploration at the same time and ensures local search and global search. Harris Hawks Optimizer (HHO) [37] is a popular population-based nongradient optimization algorithm, which has many active time varying exploration and development stages. It has strong global searching ability.

We only analyzed the possibilities of the above computational intelligence algorithms in reinforcement learning applications, but these algorithms are not really used in reinforcement learning. Therefore, in the future work, we will devote ourselves to applying computational intelligence algorithms to strategy optimization, exploration enhancement, and acceleration of learning speed in reinforcement learning.

## Figures and Tables

**Figure 1:** The update process of critic networks in DEPRL.

**Figure 2:** The framework of DEPRL.

**Figure 3:** MuJoCo test environments. (a) Hopper-v2, (b) HalfCheetah-v2, (c) Ant-v2, and (d) Walker2d-v2.

**Figure 4:** Results of each algorithm in MuJoCo test environment. (a) Hopper-v2. (b) HalfCheetah-v2. (c) Ant-v2. (d) Walker2d-v2.

**Algorithm 1:** DEPRL.

**Table 1:** The test environment in the MuJoCo benchmark.

Environment	Action dimension/state dimension	Task goals
Hopper-v2	3/11	Make a two-dimensional one-legged robot hop forward as fast as possible
HalfCheetah-v2	6/17	Make the 2D cheetah robot run fast
Ant-v2	8/111	Make a four-legged creature walk forward as fast as possible
Walker2d-v2	6/17	Make a two-dimensional bipedal robot walk forward as fast as possible

**Table 2:** Values of hyperparameter.

Hyperparameter	Values
Critic/actor learning rate	0.0003
Critic/actor hidden layer	2
Number of neurons	400/300
Critic activation	Relu
Actor activation	Tanh
Discount factor	0.99
Optimizer	Adam
Soft update coefficient	0.005
Experience pool capacity	10^6^
Experience pool sample size	100
Gauss noise	Clip ((0, 0.2), −0.5, 0.5)

**Table 3:** The mean and standard deviation of the cumulative return per turn in different MuJoCo tasks.

Task	TD3	Multiactor TD3	CEM	CEM-TD3	DPERL
Hopper-v2	3025 ± 577	3241 ± 363	1054 ± 17	3652 ± 116	3732 ± 106
HalfCheetah-v2	10002 ± 930	10341 ± 578	2298 ± 690	10978 ± 758	11615 ± 464
Ant-v2	3618 ± 425	3881 ± 319	845 ± 52	4037 ± 466	4852 ± 317
Walker2d-v2	4399 ± 238	4470 ± 301	743 ± 225	4612 ± 357	5001 ± 562

## Data Availability

The data used to support the findings of this study are available from the first author upon request.
